# *Katsuwonus pelamis* Peptide and its Complexes Protect Zebrafish and Mice From Hyperuricemia Through Promoting Kidney Excretion of Uric Acid and Inhibiting Liver Xanthine Oxidase Activity

**DOI:** 10.3389/fchem.2022.924371

**Published:** 2022-06-28

**Authors:** Wei Wei, Li-Jian Zhou, Shue Wang, Zheng Zhang, Jia-Ying Huang, Zhao Zhang, Xi-Ping Zhang, Xue-Jun Zhang, Jie Li, Ye-Wang Zhang

**Affiliations:** ^1^ School of Pharmacy, Jiangsu University, Zhenjiang, China; ^2^ The People’s Hospital of Danyang, Danyang, China; ^3^ School of Public Health, Shandong University, Jinan, China; ^4^ Zhongshiduqing Biotechnology Co., Ltd., Heze, China

**Keywords:** *Katsuwonus pelamis* peptide, *Katsuwonus pelamis* peptide complexes, zebrafish, mice, hyperuricemia

## Abstract

*Katsuwonus pelamis* peptide and its complexes have the effect of lowering uric acid (UA)-levels. To identify the effect and possible mechanisms, different concentrations of *Katsuwonus pelamis* peptide and its complexes were administered to the zebrafish and mice hyperuricemia models, and the UA level was measured. Meanwhile, the hyperuricemic mice were treated orally at 0.83, 1.67, and 5.00 mg/g body weight for 7 days with *Katsuwonus pelamis* peptide and the complexes groups, separately. The levels of serum UA (SUA), urinary UA (UUA), serum creatinine (SCR), blood urine nitrogen (BUN), and xanthine oxidase (XOD) activities were detected in each group. The results showed that the *Katsuwonus pelamis* peptide (125 μg/ml) and its complexes (83.3 and 250 μg/ml) effectively reduced UA level in zebrafish with hyperuricemia (*p* < 0.05). The *Katsuwonus pelamis* peptide at high concentration (5.00 mg/g) decreased the SUA level, SCR level, BUN level, and hepatic XOD activity, and the complexes (1.67 and 5.00 mg/g) significantly reduced the SUA level and hepatic XOD activity (*p* < 0.05) in the hyperuricemic mice. In addition, in a hyperuricemic mouse model, the UUA level was increased after treatment with *Katsuwonus pelamis* peptide and its complexes at high concentrations (*p* < 0.05). The total therapeutic effects in the *Katsuwonus pelamis* peptide complex group were better than those in the *Katsuwonus pelamis* peptide group. Thus, *Katsuwonus pelamis* peptide and its complexes may possibly be used to prevent hyperuricemia *via* promoting urate secretion and inhibiting XOD activity production.

## Introduction

Hyperuricemia is a metabolic disease with a high blood uric acid (UA) level (Eun et al., 2020; Lai et al., 2020). In the case of chronic hyperuricemia, UA is deposited in the joints in the form of monosodium urate, which is closely related to gout (Yang et al., 2018; An et al., 2020). As the important enzyme in purine metabolism in the liver, xanthine oxidase (XOD) could catalyze purine to uric acid (Huang et al., 2018; Cicero et al., 2021a). Therefore, reducing XOD activity has a prominent effect on treating hyperuricemia (Wang et al., 2018; Zhu et al., 2018; Yang et al., 2019). The current drugs for hyperuricemia, such as allopurinol (an XO inhibitor), mainly inhibit the production or promote the excretion of UA (Borghi et al., 2020), but in view of some serious side effects of these drugs, such as hypersensitivity syndrome, gastrointestinal reactions, and kidney function damage, which have been limited to long-term use (Borghi et al., 2020; Liu et al., 2020). Therefore, the development of more safer and effective drugs for treating hyperuricemia and gout is very important.

Nowadays, a growing number of natural products and their extracts have been demonstrated effective in the treatment of hyperuricemia (Zhang et al., 2019; Cicero et al., 2021b; Shi et al., 2022), which may reduce serum UA level and the occurrence of adverse reaction and need further research (Zhu et al., 2021). *Katsuwonus pelamis*, also known as bullet mackerel, is a kind of tuna with the largest amount of fish trawling in China (Yang et al., 2016; Ma et al., 2017; Weng et al., 2019). The peptide extracted from *Katsuwonus pelamis* is rich in carnosine and anserine, which would decrease UA levels effectively (Han et al., 2021). In addition, previous research has shown that *Katsuwonus pelamis* peptide contains imidazole compounds, and the molecules are very effective in lowering UA (Kubomura et al., 2016). However, the antihyperuricemia effect of *Katsuwonus pelamis* peptide has rarely been studied *in vivo*.

In this study, we identified the effects of *Katsuwonus pelamis* peptide and its complexes on reducing UA level in zebrafish and mouse hyperuricemia models. We found that *Katsuwonus pelamis* peptide and its complexes could be potential therapeutics for hyperuricemia by suppressing XO activity and promoting kidney excretion of UA.

## Materials and Methods

### Chemicals

*Katsuwonus pelamis* peptide was obtained by hydrolyzing *Katsuwonus pelamis* with protease, and *Katsuwonus pelamis* peptide complexes comprised 5% pueraria root powder, 3% coix seed, 3% galangal, 5% chrysanthemum, and 84% *Katsuwonus pelamis* peptide. Both *Katsuwonus pelamis* peptide and *Katsuwonus pelamis* peptide complexes were supplied from Zhongshiduqing Biological Co., Ltd. (Heze, China); potassium oxonate (97%) and allopurinol (≥99%) were purchased from Beijing Solabao Technology Co., Ltd. (Beijing, China); uric acid (UA), serum creatinine (SCR), blood urine nitrogen (BUN) and xanthine oxidase activity assay kits were purchased from Ningbo Meikang Biotechnology Co., Ltd. (Zhejiang, China); All the other agents were bought from Sigma-Aldrich.

### Animals and Maintenance

Two kinds of animal experimental models were used in this study: 1) Adult AB strain zebrafish were purchased from Hangzhou Huante Biological Technology Co., Ltd. All the animals were raised at the conditions including temperature (27–29°C) and pH (6.9–7.2), and salinity was strictly controlled. The male and female zebrafish were housed in a 2:2 mix in lattice containers to prevent the predation of eggs after the embryos were acquired. The age of fertilized embryos was expressed in hours (hpf) and days (dpt). 2) Eight-week-old C57BL/6 male mice were purchased from Jinan Pengyue Co., Ltd. The mice were fed under standard conditions: room temperature (24–26°C) and humidity of 50 ± 5%, allowing free access to water and food under 12 h light/dark cycle.

### Determination of MTC for *Katsuwonus pelamis* Peptide and its Complexes in Zebrafish With Hyperuricemia

The uricase inhibitor potassium oxonate was applied to induce a zebrafish hyperuricemia model. 360 hyperuricemic wild-type AB zebrafish were transferred into a six-well microplate at 3 ml/30 zebrafish volume, and they were treated with *Katsuwonus pelamis* peptide and *Katsuwonus pelamis* peptide complexes at different concentrations for 24 h. In the tests, five concentrations (125, 250, 500, 1000, and 2000 μg/ml) were used, and the mortality and toxicity were recorded at the end of the treatment. Dead zebrafish were identified with the absence of heartbeat under a dissecting stereomicroscope. The MTC of a testing drug was a maximum concentration that did not produce any observable adverse effects in hyperuricemia zebrafish models. After determining the MTC, three testing concentrations, high (MTC), medium (1/3 MTC), and low (1/9 MTC), were selected for further work.

### Assessment of *Katsuwonus pelamis* Peptide and its Complex Effects on Zebrafish With Hyperuricemia

In this work, 270 wild-type AB zebrafish with hyperuricemia were dispensed into 6-well plates in 3 ml of fish-culturing water, and potassium oxonate was used to develop zebrafish hyperuricemia models. The effects of *Katsuwonus pelamis* peptide and its complexes on hyperuricemia were assessed in these models. The zebrafish were treated with *Katsuwonus pelamis* peptide (at three concentrations: 13.9, 41.7, and 125 μg/ml) and *Katsuwonus pelamis* peptide complexes (at three concentrations: 27.8, 83.3, and 250 μg/ml) for 24 h, separately. The hyperuricemia zebrafish model only treated with xanthine sodium salt served as a hyperuricemia model, and the zebrafish with hyperuricemia treated with 136 μg/ml allopurinol were used as a positive control.

The treated zebrafish were randomly selected and set in a 96-well plate with three zebrafish per well in 50 μl uric acid detection kit solution. UA was measured by the AmplexTM Red Uric Acid/Uricase Assay Kit. The fluorescence intensity (S) was quantified in a multifunctional microplate reader, at the excitation range of 530–560 nm. During each determination, for each dose, at least six wells per sample were measured, and the results were averaged.

### Effects of *Katsuwonus pelamis* Peptide and its Complexes on the Serum UA, Serum Creatinine, Blood Urine Nitrogen, and Urinary UA Levels in Hyperuricemic Mice

Ninety mice were randomly divided into nine groups, including the control group, hyperuricemia group, allopurinol group, *Katsuwonus pelamis* peptide groups (0.83, 1.67, and 5.00 mg/g), and *Katsuwonus pelamis* peptide complex groups (0.83, 1.67, and 5.00 mg/g) (*n* = 10). Except for the control group, the other eight groups were intraperitoneally injected with potassium oxonate (250 mg/kg) at 9:00 am for 7 consecutive days. The corresponding group was orally administered with allopurinol, *Katsuwonus pelamis* peptide, and its complexes for 7 consecutive days at 2:00 pm. After the last administration on the 7th day, whole blood from each mouse was collected and centrifuged at 4000 × g for 10 min to collect the serum. Urine was collected from the mice with plastic wrap in the feeding cages. Subsequently, the collected mouse serum and urine samples were used to detect the serum UA (SUA), SCR, BUN, and urinary UA (UUA) levels according to the instructions.

### Effects of *Katsuwonus pelamis* Peptide and its Complexes on Xanthine Oxidase Activities in the Liver of Mice With Hyperuricemia

After collecting the serum and urine, the livers of the killed mice were obtained. The liver tissue of the mice was homogenized thoroughly in sodium phosphate buffer under the ice bath. The homogenate was centrifuged at 4000 × g for 20 min to collect the supernatant. The hepatic XOD activity was determined using the xanthine oxidase activity assay kit according to the instructions.

### Data Analysis

The data were analyzed by SPSS 21 software, and all data were presented as the form of $\bar{x}$ ± s. As for the data of different treatment groups, one-way ANOVA was used for analysis and comparison. The two groups were compared *via* the T test, and the test standard was α = 0.05 (bilateral).

## Results

### MTC of *Katsuwonus pelamis* Peptide and its Complexes

In the hyperuricemia zebrafish treated with *Katsuwonus pelamis* peptide 125 μg/ml, no abnormalities were observed, while 20% (6/30), 60% (18/30), 87% (26/30), and 100% (30/30) zebrafish died when treated at the concentrations of 250, 500, 1000, and 2000 μg/ml. As for *Katsuwonus pelamis* peptide complexes, there was no significant difference in the hyperuricemia zebrafish at the concentration of 125 and 250 μg/ml. Based on these results, the MTC of *Katsuwonus pelamis* peptide was determined at 125 μg/ml, and the MTC of *Katsuwonus pelamis* peptide complexes was identified at 250 μg/ml (Table 1).

**TABLE 1:** Death number and phenotypes in the zebrafish treated with *Katsuwonus pelamis* peptide and its complexes (*n* = 30).

Group	Concentration (μg/ml)	Death number (N)	Mortality (%)	Phenotypes
Normal	—	0	0	No observable abnormality
Model	—	0	0	No observable abnormality
*Katsuwonus pelamis* peptide	125	0	0	No observable abnormality
	250	6	20	—
	500	18	60	—
	1000	26	87	—
	2000	30	100	—
*Katsuwonus pelamis* peptide complexes	125	0	0	No observable abnormality
	250	0	0	No observable abnormality
	500	3	10	—
	1000	7	23	—
	2000	10	33	—

### *Katsuwonus pelamis* Peptide and its Complexes Reduced Uric Acid Level in Zebrafish With Hyperuricemia

Compared with the control group, the UA level in the model group increased (*p* < 0.05), indicating that the zebrafish model of hyperuricemia was successfully established. *Katsuwonus pelamis* peptide at a concentration of 125 μg/ml and *Katsuwonus pelamis* peptide complexes at a concentration of 250 μg/ml markedly reduced UA level in zebrafish with hyperuricemia (*p* < 0.05). In addition, the effect of lowering UA in the *Katsuwonus pelamis* peptide complex group was better than that in the *Katsuwonus pelamis* peptide group.

### *Katsuwonus pelamis* Peptide and its Complexes Regulated the Serum UA, Serum Creatinine, Blood Urine Nitrogen, and Urinary UA Levels in Mice With Hyperuricemia

After intraperitoneal injection of potassium oxonate into mice, the level of SUA in the model group was significantly higher than that of the control (*p* < 0.05), indicating that the hyperuricemia mouse model was successfully constructed (Figure 1). The SUA level in the allopurinol group was lower than that in the model group (*p* < 0.05). There was only a significant difference in the SUA level between the model group and the high concentration group of *Katsuwonus pelamis* peptide (*p* < 0.05). In the *Katsuwonus pelamis* peptide complex groups, the SUA level was also decreased (*p* < 0.05) and correlated with the concentration of the complexes. Meanwhile, there was no significant difference between the 0.83 mg/g complex group and the model group, indicating that *Katsuwonus pelamis* peptide complexes reduced the SUA level in a dose-dependent manner in mice with hyperuricemia. Simultaneously, we tested the levels of SCR and BUN. The levels of SCR and BUN decreased in both the high concentration of *Katsuwonus pelamis* peptide group and the high concentration of *Katsuwonus pelamis* peptide complex group (*p* < 0.05). In addition, compared to the model group, the levels of UUA in the *Katsuwonus pelamis* peptide (5.00 mg/g) group and complex (5.00 mg/g) group were increased (*p* < 0.05) (Figure 2). Thus, *Katsuwonus pelamis* peptide and its complexes reduced the SUA levels in hyperuricemic mice and were likely to increase the excretion of UA from blood to urine. Also, our results showed that *Katsuwonus pelamis* peptide and its complexes have no apparent effect on the body weight of the mice (the data were not shown).

**FIGURE 1:** Effect of *Katsuwonus pelamis* peptide and its complexes on the UA content in potassium oxonate–induced hyperuricemic zebrafish. ^#^ *p* < 0.05 compared with the control group; *p < 0.05 compared with the model group.

**FIGURE 2:** Effect of *Katsuwonus pelamis* peptide and its complexes on the SUA level, SCR level, BUN level, and UUA level of potassium oxonate–induced hyperuricemic mice. ^#^ *p* < 0.05 compared with the control group; *p < 0.05 and **p < 0.01 compared with the model group.

### *Katsuwonus pelamis* Peptide and its Complexes Suppress Hepatic Xanthine Oxidase Activities in the Mice With Hyperuricemia

Further experiments were performed to check whether *Katsuwonus pelamis* peptide and its complexes reduce SUA levels in hyperuricemic mice. Compared with the control group, the hepatic XOD activity of the model group was significantly increased (*p* < 0.5). Also, the hepatic XOD activity of the allopurinol group was obviously restrained compared to that of the model group (*p* < 0.05). The hepatic XOD activities in the *Katsuwonus pelamis* peptide groups were lower than those of the model group, but there was a significant difference in hepatic XOD activity between the model group and the high-concentration group of *Katsuwonus pelamis* peptide (*p* < 0.05). In the *Katsuwonus pelamis* peptide complex (1.67 and 5.00 mg/g) groups, the hepatic XOD activities were also inhibited compared to those in the model group (*p* < 0.05) (Figure 3). The results indicated that the potential mechanism of lowering SUA was by suppressing XOD activity.

**FIGURE 3:** Effects of *Katsuwonus pelamis* peptide and its complexes on hepatic XOD activities in hyperuricemic mice induced by potassium oxonate. ^#^ *p* < 0.05 compared with the control group; *p < 0.05 compared with the model group.

## Discussion

Hyperuricemia is a metabolic disease caused by disturbances in UA metabolism, which would cause gouty arthritis, systemic inflammation, renal insufficiency, and other metabolic abnormalities (Hu and Brown, 2020; Li et al., 2020; Cicero et al., 2021b). Hyperuricemia is due to insufficient UA excretion by the kidney and excessive UA production by the liver. The overproduction of UA is mainly caused by increased activity of the key enzyme XOD during the production of UA (Niu et al., 2017; Wang et al., 2021a). Therefore, it is essential to regulate XOD activity in the liver for hyperuricemia treatment.

Benzbromarone, a clinical first-line anti-hyperuricemia drug, plays the role of maintaining blood UA at an appropriate level *via* enhancing UA excretion in the proximal tubules of the kidney (Wang et al., 2021b; Liu et al., 2021). Nevertheless, numerous studies have demonstrated that benzbromarone is hepatotoxic, which has limited its use in the United States and some other countries (Nakata et al., 2020). Allopurinol, another clinical treatment for hyperuricemia, decreases hepatic UA production primarily by inhibiting the activity of XOD (Hu and Brown, 2020; Floege and Johnson, 2021). However, studies have suggested that serious side effects may occur after taking the drug. Hence, there is an urgent need to develop new antihyperuricemia drugs.

*Katsuwonus pelamis* is one of the important commercial species, growing globally at more than 3 million tons per year. In China, numerous fish by-products are produced during the *Katsuwonus pelamis* can production, such as bioactive peptides, collagen, and gelatin (Qiu et al., 2019). *Katsuwonus pelamis* peptide has protective effects on liver and kidney tissue (Kubomura et al., 2016; Al-Najjar et al., 2019; Pragnya et al., 2020). However, the effect of *Katsuwonus pelamis* peptide on hyperuricemia is still unclear.

In this study, we found that *Katsuwonus pelamis* peptide (125 μg/ml) and *Katsuwonus pelamis* peptide complexes (250 μg/ml) effectively reduced UA levels in the zebrafish with hyperuricemia. In hyperuricemia mouse models, the treatments with *Katsuwonus pelamis* peptide and its complexes at a high concentration (5.00 mg/g) decreased the SUA level, SCR level, BUN level, and hepatic XOD activity, indicating the protective effect on the kidney. Some studies have found that the peptide extracted from *Katsuwonus pelamis* could strengthens the anti-inflammatory and regulates intestinal flora (Kang et al., 2016; Chansuwan et al., 2019; Wang et al., 2019). These findings may explain why *Katsuwonus pelamis* peptide and its complexes possess the ability to inhibit XOD activity. However, further verification is still needed. In addition, after being treated with *Katsuwonus pelamis* peptide and its complexes, the UUA level in hyperuricemic mice was increased, which revealed that the decrease in SUA was related to increased UUA excretion.

The natural peptide extracted from *Katsuwonus pelamis* lowered UA levels in zebrafish and mice with hyperuricemia, mainly by inhibiting XOD activity and promoting urate secretion. *Katsuwonus pelamis* peptide may have great potential for prevention and treatment of hyperuricemia.

## Data Availability

The original contributions presented in the study are included in the article/Supplementary Material; further inquiries can be directed to the corresponding author.
